This article has been retracted.

# SDTM: A Novel Topic Model Framework for Syndrome Differentiation in Traditional Chinese Medicine

**DOI:** 10.1155/2022/6938506

**Published:** 2022-01-04

**Authors:** Jialin Ma, Xiaoqiang Gong, Zhaojun Wang, Qian Xie

**Affiliations:** ^1^Jiangsu Internet of Things and Mobile Internet Technology Engineering Laboratory, Huaiyin Institute of Technology, Huaian 223003, China; ^2^AVIC Xi'an Aircraft Industry Group Company Ltd., Xi'an 710089, China; ^3^Huaiyin Wu Jutong Institute of Traditional Chinese Medicine, Huaian 223000, China; ^4^Jiangsu Eazytec Co. Ltd., Wuxi, China

## Abstract

Syndrome differentiation is the most basic diagnostic method in traditional Chinese medicine (TCM). The process of syndrome differentiation is difficult and challenging due to its complexity, diversity, and vagueness. Recently, artificial intelligent methods have been introduced to discover the regularities of syndrome differentiation from TCM medical records, but the existing DM algorithms failed to consider how a syndrome is generated according to TCM theories. In this paper, we propose a novel topic model framework named syndrome differentiation topic model (SDTM) to dynamically characterize the process of syndrome differentiation. The SDTM framework utilizes latent Dirichlet allocation (LDA) to discover the latent semantic relationship between symptoms and syndromes in mass of Chinese medical records. We also use similarity measurement method to make the uninterpretable topics correspond with the labeled syndromes. Finally, Bayesian method is used in the final differentiated syndromes. Experimental results show the superiority of SDTM over existing topic models for the task of syndrome differentiation.

## 1. Introduction

As an important complementary medical system to modern biomedicine, traditional Chinese medicine (TCM) has played an indispensable role in healthcare of Chinese people for several thousand years [1, 2]. In recent years, the TCM has become more and more popular all over the world [3]. Doctors usually adopt four diagnostic ways to obtain symptoms, that is, observation, listening, interrogation, and pulse-taking in TCM [4]. A syndrome can be summarized via a set of symptoms, which are intrinsically related to each other. This process is the key to differentiating syndromes. An example of syndrome is given in Figure 1, which is selected from [4]. It includes syndrome name, symptoms, pathogenesis, treatment, representative prescription, and common medicines [5–7].

One of the significant characteristics of TCM is to treat diseases based on syndrome differentiation. This is a process of comprehensive judgment based on analysis, induction, and reasoning via four-way information diagnosis [8]. This is also the key link for doctors to select proper prescriptions or therapies. Syndrome differentiation is a process through which doctors make a diagnosis based on subjective knowledge and experience in accord with the objective reality of a patient. Because of the differences in individuals and the limited knowledge or experience of doctors, one patient may be diagnosed with different syndromes by different doctors [9].

In order to accurately master the complex structure of syndromes and establish a diagnostic standard for TCM, in time, it is of great significance to analyze the principles of syndrome differentiation. This is beneficial for the inheritance, the improvement, and the development of the diagnosis theory of TCM [10–12].

In the long Chinese history, a large number of medical records were recorded in ancient textbooks or hospitals, which include abundant knowledge and experience about TCM diagnose. Therefore, mass of TCM knowledge is hidden in these medical records. Data mining is an important technology to discover hidden knowledge from large-scale data [13–15]. However, TCM medical records are often represented by text documents, as shown in Figure 2, in which TCM knowledge is characterized by natural language. Although the semantic understanding has made great progress in the field of artificial intelligence in recent years, and some methods have been proposed to assist physicians in decision-making by mining medical records, they failed to comprehensively describe how a syndrome is generated according TCM theories [16–19].

Topic model is an effective statistical model for discovering the abstract topics hidden in documents, and a topic is an abstract concept, which is composed of some semantically related words [20]. Although the model has been successfully applied to latent semantic analysis and knowledge discovery, such as topic discovery, emotion analysis, and even image analysis, how to effectively integrate the actual theory of analysis objects is the key. Therefore, we adopt the topic model to capture the principles of TCM syndrome differentiation [21–23].

For syndrome differentiation in TCM, we can regard a medical record as a “document” (a group of symptoms) and syndromes in medical records as “topics.” Topic models such as PLSA and LDA are successful at discovering hidden topics from a large scale of documents, but when they are used to discover syndrome regularities, the extracted topics have low interpretability; that is, topic labels inferred from the first few words in the topic may be incorrect, because these words may not be related to the topic. Moreover, these topic models can only discover the semantic relationship between symptoms and syndromes but cannot independently characterize how a syndrome is generated using TCM theories [24–26].

In this paper, we propose a novel topic model framework to dynamically characterize the process of syndrome differentiation of TCM. The overall framework of the SDTM is shown in Figure 3. First, we propose a novel LDA-based model approach to discover the latent semantic relationship between symptoms and syndromes in Chinese medical records. Then, the corresponding syndromes are labeled for these topics based on similarity measurement in order to improve interpretability of topics. Finally, we utilize Bayesian method to implement syndrome differentiation. Our method contributes to a better understanding of TCM diagnostic principles and provides an effective model for computer automatic diagnosis.

The rest of this paper is organized as follows: Section 2 reviews some related works.  Section 3 shows the specific differentiation process of syndromes. The experimental results are analyzed in Section 4. Finally, conclusion and future work are given in Section 5.

## 2. Related Works

### 2.1. TCM Knowledge Discovery

Knowledge discovery and data mining have become popular topics in healthcare and biomedicine [27]. The research of TCM knowledge discovery is summarized by Feng et al. [21], Lukman et al. [22], Wu et al. [23], and Liu et al. [27]. Many methods have been proposed to discover some regularities in TCM diagnosis and treatments. Zhang et al. [13] proposed a novel method based on author-topic model, called the symptom-herb-diagnosis topic model (SHDTM), to automatically extract the relationships between symptoms, herb groups, and diagnoses from TCM clinical data. Erosheva et al. [14] used link latent Dirichlet allocation (LinkLDA) to extract the latent topics with both symptoms and their corresponding herbs in clinical cases. Yao et al. [1] applied LDA and TCM domain knowledge to mine treatment patterns in TCM clinical cases.

### 2.2. Topic Model

Recently, topic model, as a popular text analysis method, can detect latent topics in large-scale documents [24]. It is known that two classical topic models have been extensively applied to document analysis. They are probabilistic latent semantic analysis (PLSA) and latent Dirichlet allocation (LDA) [25]. In PLSA, a document is regarded as a mixture of topics, where a topic is determined by the probability distribution over words. In order to solve the limitation of PLSA, LDA adds Dirichlet priors in the distributions; it is a complete generative model and achieves great successes in text mining. Moreover, LDA can also be utilized in the tasks of health and biomedicine mining [13, 27–30]. For instance, Yao et al. [15] discovered some important treatment patterns in TCM clinical cases by exploiting the supervised topic model and domain knowledge. Chen et al. [20] demonstrated that the configuration of functional groups in metagenome samples can be inferred by probabilistic topic model. Huang et al. [29] mined the latent treatment patterns for clinical pathways through topic model. In addition, some improved topic models are also proposed for short texts analysis, such as author-topic model (ATM) [26] and block-LDA [30].

However, a standard LDA still cannot be directly used for TCM mining, because it is an unsupervised topic model, which is unable to express the relationships between syndromes and symptoms [31–33]. Furthermore, the abovementioned research failed to consider the syndrome differentiation principles [34–38]. Therefore, we propose a novel topic model framework called syndrome differentiation topic model to dynamically characterize the process of TCM syndrome differentiation.

## 3. Method

In this section, we present the framework named SDTM to characterize how a syndrome is generated according to TCM theory. It consists of three steps: topic modeling of Chinese medical records, syndrome labeling, and syndrome differentiation.

### 3.1. Topic Modeling of Chinese Medical Records

In the process of diagnosis and treatment, the TCM doctors usually obtain symptoms through four diagnostic ways, i.e., observation, listening, interrogation, and pulse-taking, and then infer syndrome differentiation for patient according TCM theories. It is a complicated process that relies on the experience and knowledge of the doctor. To explore the problem, an LDA-based method is developed to discover the latent semantic relationships between symptoms and syndromes by medical records. We use the topic model LDA to model the above process of syndrome inferring.

#### 3.1.1. Model Generative Process

The graphical representation of topic modeling of Chinese medical records is given in Figure 4. The meaning of notations is illustrated in Table 1.

When modeling the Chinese medical records in the frame SDTM, let *M* be the number of medical records, where each medical record *m* owns *N*_*s*_*m*__ symptoms, *s*_*mn*_ is the *n*th symptom in medical record *m*, and *z*_*mn*_ (*n*=1,  2,   ⋯ ,  *N*) is the latent syndrome distribution for *s*_*mn*_. For instance, the medical record in Figure 2 has *N*_*s*_*m*__ = 18 symptoms, and the latent syndrome distribution for the symptom “diuresis” should be “two deficiency syndrome of liver and kidney” or “syndrome of dampness-heat blocking collaterals.” Let *K* be the number of topics, a topic *k*∫{1,  2,   …,  *K*} represent a syndrome, and *φ*_*k*_ be the *N*-dimensional syndrome-symptom multinomial for syndrome *k*, where *N* is the number of all unique symptoms in *M* medical records. *θ*_*m*_ is the *K*-dimensional medical record-syndrome multinomial for medical record *m*. *α* and *β* are the hyperparameters of the Dirichlet priors on *θ*_*m*_ and *φ*_*k*_, respectively.

The modeling process of Chinese medical records is given as follows:

(1) For syndrome *k* in 1,  2,   …,  *K*, draw *φ*_*k*_ ~ Dir(*β*).
(2) For medical record *m*, draw *θ*_*m*_ ~ Dir(*α*).
(3) For each of the *N*_*s*_*m*__ symptoms in medical record *m*:
  - Draw a syndrome *z*_*mn*_ ~ Mult(*θ*_*m*_).
  - Draw a symptom *s*_*mn*_ ~ Mult(*φ*_*k*_).

Here, Dir is a convenient distribution on the simplex. It is in the exponential family and has finite dimensional sufficient statistics. It is conjugate to the multinomial distribution [9]. Mult represents the multinomial distribution.

#### 3.1.2. Model Inference and Learning

Gibbs sampling is an effectively and widely used Markov chain Monte Carlo algorithm for latent variable inference [24, 25]. We use Gibbs sampling to extract latent syndrome distributions *z*_*mn*_; it is defined as follows:

(1) $$\begin{array}{c} p\left(\;z_{mn}=k|s_{mn},s_{-mn},\;z_{-mn},z,\alpha ,\beta \right)\\ \propto \frac{n_{m}^{k}+\alpha }{\sum_{k=1}^{k}n_{m}^{k}=K\alpha }\times \frac{n_{k}^{s_{mn}}+\beta }{\sum_{i=1}^{N}n_{k}^{s_{i}}=N\beta }, \end{array}$$

where *k* represents a syndrome, *s*_−*mn*_ represents all symptoms except *s*_*mn*_, *z*_−*mn*_ represent the syndrome distributions for all symptoms except *s*_*mn*_, *z* represent the syndrome distributions for all symptoms, *n*_*m*_^*k*^ is the number of times syndrome *k* occurs in medical record *m*, and *n*_*k*_^*s*_*mn*_^ is the number of times *s*_*mn*_ is assigned to syndrome *k*.

According to Gibbs sampling, *θ*_*m*_ and *φ*_*k*_ can be calculated as follows:

(2) $$\begin{array}{c} \theta_{m}\left(k\right)=\frac{n_{m}^{k}+\alpha }{\sum_{K=1}^{K}n_{m+K\alpha }^{k}},\\ \;\varphi_{k}\left(s_{mn}\right)=\frac{n_{k}^{s_{mn}}+\beta }{\sum_{i=1}^{N}n_{k}^{s_{i}}+N\beta }. \end{array}$$

### 3.2. Syndrome Labeling

Although topic modeling of Chinese medical records is successful in discovering hidden topics from medical records, each of these topics lacks an identifiable label, which results in low interpretability. Therefore, to improve the interpretability of topics, we label a syndrome on each topic by mapping symptoms in a topic to syndromes in TCM domain. First, we select data from [4] to build a standard syndrome database with *d* syndromes. Then syndrome *y*_*j*_ (*j*∫[1,  2,   …, *d*]) in the syndrome database is assigned to topic *k*∫[1,  2,   …,  *K*] based on the similarity between *k* and *y*_*j*_, which is calculated using Jaccard similarity coefficient as follows [25]:

(3) $$\begin{array}{c} \underset{\;j\text{Î}\left[1,2,L,d\right]}{y=\arg\;\max}\text{sim}\left(k,y_{j}\right)=\underset{j\text{Î}\left[1,2,L,d\right]}{\arg\;\max}\frac{\left|kÇy_{j}\right|}{\left|k\text{È}y_{j}\right|}, \end{array}$$

where *d* is the number of syndromes in standard syndrome database and *y*_*j*_ represents the *j*th syndrome in the standard syndrome database.

### 3.3. Syndrome Differentiation

After these syndromes are assigned, probability $p\left(k|\overset{⟶}{H\left(s\right)}\right)$ of syndrome (topic) *k* for medical record $\overset{⟶}{H\left(s\right)}$ can be computed using the Bayesian formula as follows:

(4) $$\begin{array}{c} p\left(k\overset{⟶}{H\left(s\right)}\right)\propto \frac{\sum_{s_{i}\in \overset{⟶}{H\left(s\right)}}p\left(s_{i}|k\right)p\left(k\right)}{\left|\overset{⟶}{H\left(s\right)}\right|}\\ =\;\frac{\sum_{s_{i}\in \overset{⟶}{H\left(s\right)}}\;\varphi_{k}\left(s_{i}\right)p\left(k\right)\left(k\right)}{\left|\overset{⟶}{H\left(s\right)}\right|}\propto \frac{\sum_{s_{i}\in \overset{⟶}{H\left(s\right)}}\varphi_{k}\left(s_{i}\right)}{\left|\overset{⟶}{H\left(s\right)}\right|}, \end{array}$$

where a new medical record is represented by a set of symptoms $\overset{⟶}{H\left(s\right)}$, $p\left(k|\overset{⟶}{H\left(s\right)}\right)$ is the probability of syndrome *k* given medical record $\overset{⟶}{H\left(s\right)}$, *p*(*s*_*i*_*|k*) is the probability of symptom *s*_*i*_ given syndrome *k* which is equal to  *φ*_*k*_(*s*_*i*_), *p*(*k*) is the prior of syndrome *k* which can be regarded as a constant, and $\left|\overset{⟶}{H\left(s\right)}\right|$ is the number of symptoms in the new medical record $\overset{⟶}{H\left(s\right)}$.

To differentiate the syndromes for a given medical record, we exploit the symptom vector to represent the medical record:

(5) $$\begin{array}{c} \;\overset{⟶}{H\left(s\right)}=\left(s_{1},\ldots ,s_{i},\ldots ,s_{n}\right), \end{array}$$

where symptom *s*_*i*_ is a binary indicator; if a medical record contains *s*_*i*_, it is equal to 1; otherwise, it equals 0.

We take the posterior vector as the feature vector of medical record $\overset{⟶}{H\left(s\right)}$:

(6) $$\begin{array}{c} \theta_{\overset{⟶}{H\left(s\right)}}=\left\{p\left(1|\overset{⟶}{H\left(s\right)}\right),\ldots ,p\left(i|\overset{⟶}{H\left(s\right)}\right),\ldots ,p\left(K|\overset{⟶}{H\left(s\right)}\right)\right\}, \end{array}$$

where $p\left(i|\overset{⟶}{H\left(s\right)}\right)$ represents the probability of syndrome *i* which is calculated via (4).

We use (6) to determine syndromes of medical record $\overset{⟶}{H\left(s\right)}$:

(7) $$\begin{array}{c} {\text{Syndrome}}_{\overset{⟶}{H\left(s\right)}}=\left\{k|p\left(k|\overset{⟶}{H\left(s\right)}\right)>T,\;k\in 1,2,\ldots ,K,\overset{⟶}{H\left(s\right)}\varepsilon R^{n}\right\}, \end{array}$$

where *T* is the syndrome differentiation threshold and *n* is the number of symptoms in $\overset{⟶}{H\left(s\right)}$.

## 4. Experimental Results

In the section, we evaluate our framework, SDTM, on three experimental tasks for Chinese medical records. In particular, we want to determine the following:

- Can our SDTM achieve the best generalization performance compared to other topic models?
- Can our SDTM differentiate syndromes for a set of symptoms?
- Can our model reflect the patterns of TCM syndrome differentiation?

All experiments are tested in MATLAB 2015a and implemented on a computer with Intel Core i3-7100, 3.90 GHz CPU, 8 GB RAM, and Windows 10 64-bit operating system. Each experiment is run 10 times.

### 4.1. Dataset

Chronic kidney disease (CKD) is a common condition in clinical practice. The basic clinical manifestations of the disease include proteinuria, hematuria, hypertension, and edema. The disease has insidious cause, long course, and slow change of state, so its clinical treatment is difficult. Although modern medicine has adopted such means as controlling hypertension, reducing proteinuria and lipid, the prognosis is not good. Traditional Chinese medicine has significant advantages in the treatment of the disease, such as reducing adverse drug reactions and inhibiting relapse of the disease. We collected 1959 medical records on CKD from Beijing Dongzhimen Hospital, which include 948 (48.4%) females and 1011 (51.6%) males. The dataset mainly contains 4 syndromes, i.e., “deficiency of Qi and blood,” “retention of dampness and blood stasis,” “blood stasis in collaterals,” and “retention of water in the body,” and 9 diseases, i.e., “nephrotic syndrome,” “diabetes,” “chronic nephritis,” “hypertension,” “cerebral embolism,” “hyperuricemia,” “hyperlipidemia,” “membranous nephropathy,” and “IgA nephropathy.” For example, a medical record case is shown in Figure 2, where the texts in red are considered to be the descriptions of symptoms. For each medical record, we first filter indication symptoms contained in the medical record by utilizing standard symptoms in [27] and manually remove the other elements in the medical record except symptoms and syndromes. Then, we utilize the one-hot vector to represent each medical record. Finally, we randomly select 1469 medical records as the training set and 490 medical records as the testing set.  Table 2 lists the demographic and clinical characteristics of the dataset.


(8) $$\begin{array}{c} \text{perplexity}\left(u_{\text{test}}|s_{\text{test}}\right)=\text{exp}\left(-\frac{\sum_{p=1}^{P_{\text{test}}}\log\;p\left(\overset{⟶}{u_{p}}|\overset{⟶}{s_{p}}\right)}{\sum_{p=1}^{P_{\text{test}}}N_{u_{p}}}\right)\;,\;\\ p\left(\overset{⟶}{u_{p}}|\overset{⟶}{s_{p}}\right)=\prod_{u_{pn}\in \overset{⟶}{u_{p}}}p\left(u_{pn}|\overset{⟶}{s_{p}}\right)\;=\prod_{u_{pn}\in \overset{⟶}{u_{p}}}\frac{1}{N_{s_{p}}}\sum_{s_{pl}\in \overset{⟶}{s_{p}}}p\left(u_{pn}|s_{pl}\right), \end{array}$$

### 4.2. Baselines

We compare our method with the following baselines:

1. Author-topic model (ATM) [26]: ATM is an extended LDA model, which extracts the topic distribution by utilizing the author information contained in documents. Here, we regard syndromes as authors and symptoms as words.
2. LinkLDA [28]: LinkLDA is also a probabilistic generative model, which considers both the words in documents and the reference document information of these words. Here, we regard symptoms as words and references.
3. Block-LDA [30]: Block-LDA is an extended LinkLDA model which models links between certain types of entities. Here, we regard symptoms as words and regard symptom-pair set extracted from all training medical records as the external links.
4. Symptom-syndrome topic model (SSTM): SSTM proposed in previous work [11] is an LDA-based topic model, which regards syndromes as topics and symptoms as words.

### 4.3. Evaluation Metrics

Here, we use the differentiated perplexity to evaluate the generalization performance of topic models. A lower perplexity means generalization performance of the topic model is better. The differentiated perplexity of a set of test symptoms is defined as follows [24]:where *s*_test_ are the symptoms in test medical records, *u*_test_ are syndromes in test medical records, $\overset{⟶}{s_{p}}$ are symptoms in medical record *p* of the test set, $\overset{⟶}{u_{p}}$ are syndromes in medical record *p* of the test set, *P*_test_ is the number of medical records in the test set, *N*_*u*_*p*__ is the number of syndromes in test medical record *p*, *u*_*pn*_ represents *n*th syndrome in syndromes $\overset{⟶}{u_{p}}$, and *s*_*pl*_ represents *l*th symptom in symptoms $\overset{⟶}{s_{p}}$.

The probability of a syndrome *u* given a symptom *s* is as follows [37]:

(9) $$\begin{array}{c} p\left(u|s\right)=\sum_{p}p\left(u|p\right)\sum_{k}p\left(k|s\right),\\ =\sum_{p}\theta_{p}\left(u\right)\sum_{k}\frac{\;\varphi_{k}\left(s\right)}{\sum_{p,k}\varphi_{k}\left(s\right)}\text{ .} \end{array}$$

Meanwhile, we use the accuracy to evaluate syndrome differentiated power of topic models. A higher accuracy indicates better syndrome differentiated power, which is defined as

(10) $$\begin{array}{c} \text{accuracy}=\;\frac{\left|Y\right|}{\left|{\text{Syndrome}}_{\overset{⟶}{H\left(s\right)}}\right|}, \end{array}$$

where |*Y*| is the number of true syndromes in ${\text{Syndrome}}_{\overset{⟶}{H\left(s\right)}}$.

### 4.4. Parameter Settings

For all the models in comparison, we set hyperparameters *α*=50/*K*, *β*=0.01, and the number of standard syndromes *d*=137. We use 1000 Gibbs sampling iterations to train all topic models.

For all tests, we use Jaccard similarity coefficient to measure the similarity between syndromes *X* and *X*′, which is defined as follows:

(11) $$\begin{array}{c} \text{Sim}\left(X,X^{\prime }\right)=\frac{\left|X\cap X^{\prime }\right|}{\left|X\cup X^{\prime }\right|}, \end{array}$$

where *X* represents a syndrome in a test medical record and *X*′ represents a predicted syndrome in $Syn\;dr\;ome_{\overset{⟶}{H\left(s\right)}}$.

For similarity threshold *C*, if Sim(*X*, *X*′) > *C*, then *X*′ is a true syndrome. In the stage of syndrome differentiation, we need to determine threshold *T* so that we can differentiate syndromes for each medical record. However, there is no theoretical guidance for automatically selecting an optimal threshold for syndrome differentiation. Therefore, when *K* and *C* are both fixed, we use different thresholds *T* to compare the perplexity and accuracy.

As shown in Table 3, the value of *T* has a significant influence on the syndrome differentiation results. When *T*=1*e* − 7, all methods achieve the best syndrome differentiation results, and SDTM outperforms ATM, LinkLDA, Block-LDA, and SSTM in terms of perplexity and accuracy, so we select *T*=1*e* − 7 as an optimal threshold.

In the stage of syndrome evaluation stage, we need to determine similarity threshold *C* so that we can select true syndromes from the syndromes differentiated by SDTM. Therefore, when *K* is fixed and *T*=1*e* − 7, we use different thresholds *C* to compare the accuracy of all models. As shown in Figure 5, for different models, the accuracy of syndrome differentiation varies with the value of *C*. It is clearly seen that when *C*=0.6, all models obtain the highest number of true syndromes, and SDTM substantially outperforms the other four models in terms of accuracy, so we take *C*=0.6 as an optimal similarity threshold for selecting true syndromes.

### 4.5. Experimental Results

#### 4.5.1. Generalization Performance

Figure 6 shows the variation of perplexity with the increase of topics. It is seen that the average perplexity of SDTM is less than those of the other four models. This demonstrates that our model is more efficient in the task of syndrome differentiation. When *K* is equal to 40, SDTM achieves the minimum perplexity, which means that the best generalization performance is achieved.

#### 4.5.2. Syndrome Differentiation

Figure 7 shows the variation of accuracy with increasing of topics. The average accuracy of SDTM is higher than that of the other four models in Figure 7. When *K* is equal to 40, the SDTM achieves the highest accuracy.

In summary, from Figures 6 and 7, we can see that when *K* is equal to 40, the SDTM has the best generalization performance and syndrome differentiated power, so we take *K*=40 as the optimal number of topics.

#### 4.5.3. Discovery of Syndrome Pattern

The top five topics generated by several baseline methods are shown in Tables 4–8, respectively. The top ten symptoms in each “syndrome” topic are also shown, where italicized symptoms are not related to the syndrome. Compared with the other four methods, our SDTM can discover the best differentiated results of syndromes, and most of symptoms in each “syndrome” topic can be validated effectively by the true syndromes in [4]. From Tables 4–8, we draw the following results for the discovered syndrome patterns.

The first “syndrome” topic is “two deficiency syndrome of liver and kidney.” The results are shown in Tables 1–8: (1) ATM cannot discover a good topic; only the symptoms “inhibited defecation,” “bowel 1 per day,” and “weak” are related. (2) LinkLDA discovers one topic with five related symptoms. (3) Block-LDA and SSTM discover seven related symptoms. (4) SDTM discovers a good topic with nine related symptoms.

The second “syndrome” topic is “syndrome of dampness-heat blocking collaterals.” We find the following results: (1) ATM cannot provide a good topic again; only “palpitation,” “abnormal diet,” and “dark red tongue” are related symptoms. (2) LinkLDA discovers a little better topic with four related symptoms. (3) Block-LDA and SSTM discover six related symptoms. (4) SDTM discovers eight related symptoms.

The third “syndrome” topic is “syndrome of dampness-heat diffusing downward.” We find the following results: (1) ATM discovers a little better topic with five related symptoms. (2) LinkLDA cannot discover a meaningful topic including only three related symptoms, namely, “thin fur,” “soreness of waist,” and “hard stool.” (3) Block-LDA and SSTM discover six related symptoms. (4) SDTM discovers eight related symptoms.

The fourth “syndrome” topic is “syndrome of yang deficiency of spleen and kidney.” We have the following results: (1) ATM and LinkLDA discover four related symptoms. (2) Block-LDA and SSTM discover six related symptoms. (3) SDTM discovers nine related symptoms.

The fifth “syndrome” topic is “syndrome of yin deficiency and dampness-heat.” We have the following results: (1) ATM discovers four related symptoms. (2) LinkLDA discovers only three related symptoms. (3) Block-LDA discovers five related symptoms. (4) SSTM discovers six related symptoms. (5) SDTM discovers nine related symptoms.

From the abovementioned five topics, we find that SDTM can discover “syndrome” the most related topics.

## 5. Conclusion and Future Work

We present a novel framework, SDTM, in this paper which can effectively analyze complex and changeable syndrome differentiation patterns from TCM historical clinic records. The framework SDTM conforms to the relevant theories of TCM. The experimental results on 1959 medical records show that SDTM can discover meaningful syndrome patterns and outperforms several baseline methods. Furthermore, this study provides a framework for TCM intelligent diagnosis. However, this novel model requires annotated datasets which are often difficult to obtain.

In future work, we plan to incorporate more medical information into the model in our framework, such as disease location, pathogeny, and nature of disease in order to discover more accurate syndrome patterns. In addition, the same symptom could be described by different terms in the experimental data. This may degrade the performance of our method, so we will consider adopting metric learning for normalizing symptom in medical records in the future.

## Figures and Tables

**Figure 1:** An example of syndrome case.

**Figure 2:** An example of medical record case.

**Figure 3:** The overall process of SDTM.

**Figure 4:** Graphical model representation of topic modeling for Chinese medical records.

**Figure 5:** The accuracy of syndrome differentiation for different threshold values *C* under different models (*T*=1*e* − 7).

**Figure 6:** The differentiated perplexity of syndromes for different number of topics *K* under different models (*T*=1*e* − 7,  *C*=0.6).

**Figure 7:** The differentiated accuracy of syndromes under different models for different number of topics *K* (*T*=1*e* − 7,  *C*=0.6).

**Table 1:** Mathematical notations.

Symbol	Description
*M*	The number of medical records
*K*	The number of topics (syndromes)
*N*	The number of all unique symptoms
*N*_*s*_*m*__	The number of symptoms in medical record *m*
*s*_*mn*_	The *n*th symptom in medical record *m*
*z*_*mn*_	The latent syndrome distribution for *s*_*mn*_
*θ*_*m*_	The medical record-syndrome multinomial for medical record *m*
*φ*_*k*_	The syndrome-symptom multinomial for syndrome *k*
*α*	Hyperparameter of the Dirichlet prior on *θ*_*m*_
*β*	Hyperparameter of the Dirichlet prior on *φ*_*k*_

**Table 2:** The clinical characteristics of the training dataset with CKD.

	Deficiency of Qi and blood (918)	Retention of dampness and blood stasis (639)	Blood stasis in collaterals (444)	Retention of water in the body (399)
Female (948)	507 (53.5%)	237 (25.0%)	222 (23.4%)	228 (24.1%)
Male (1011)	411 (40.7%)	402 (39.8%)	222 (22.0%)	171 (16.9%)
Nephrotic syndrome (1272)	885 (69.6%)	627 (49.3%)	330 (25.9%)	372 (29.2%)
Diabetes (426)	57 (13.4%)	12 (2.8%)	105 (24.6%)	24 (5.6%)
Chronic nephritis (300)	117 (39%)	81 (27.0%)	6 (2.0%)	6 (2.0%)
Hypertension (192)	15 (7.8%)	0	39 (20.3%)	6 (3.1%)
Cerebral embolism (174)	171 (98.3%)	42 (24.1%)	108 (62.1%)	102 (58.6%)
Hyperuricemia (102)	30 (29.4%)	51 (50.0%)	3 (2.9%)	9 (8.9%)
Hyperlipidemia (96)	6 (6.3%)	3 (3.1%)	9 (9.4%)	3 (3.1%)
Membranous nephropathy (84)	51 (60.7%)	36 (42.6%)	24 (28.6%)	15 (17.9%)
IgA nephropathy (78)	15 (19.2%)	39 (50.0%)	3 (3.8%)	6 (7.7%)

**Table 3:** Perplexity (per) and accuracy (acc) of all models with different syndrome differentiation threshold values *T*.

*T*	ATM		LinkLDA		Block-LDA		SSTM		SDTM	
	Per	Acc	Per	Acc	Per	Acc	Per	Acc	Per	Acc
1*e* − 5	475.13	0.4132	426.68	0.4504	391.45	0.5266	275.48	0.5837	242.18	0.6075
1*e* − 6	491.21	0.4930	453.73	0.5903	365.58	0.6137	231.50	0.6395	221.31	0.6724
1*e* − 7	478.33	0.5227	382.58	0.6167	374.25	0.6476	240.75	0.6824	**218.24**	**0.8014**
1*e* − 8	496.55	0.4736	396.63	0.5433	418.41	0.5822	279.63	0.6567	295.78	0.7202
1*e* − 9	548.57	0.4462	525.50	0.5067	522.65	0.5384	324.46	0.5925	430.74	0.6873

Bold numbers indicate good experimental data.

**Table 4:** Topics learned by ATM with *K*=40.

ATM				
Two deficiency syndrome of liver and kidney	Syndrome of dampness-heat blocking collaterals	Syndrome of dampness-heat diffusing downward	Syndrome of yang deficiency of spleen and kidney	Syndrome of yin deficiency and dampness-heat
Inhibited defecation	Palpitation	Soreness of waist	Sallow complexion	*Sunken pulse*
*Leg swelling*	*Knee pain*	*Dark red tongue*	*Fissured tongue*	*Debility of the legs*
*Hypermenorrhea*	*Bowel 1 per day*	Emaciation	Soreness of waist	Irritability
*Stomachache*	*Arthralgia*	*Bowel 1 per day*	*Lassitude*	*Dark red tongue*
*Phlegm yellow*	*Urine astringency*	*Nausea*	No abdominal distention	*Bowel 1 per day*
Bowel 1 per day	Abnormal diet	Thin fur	*Dark red tongue*	Brown macules on the skin
*No hard stool*	*Bowel 1 per day*	*Bodily pain*	Loose stool	No abdominal distention
Weak	Dark red tongue	Weak	*Cramp*	*Hematochezia*
*Dark red tongue*	*Weak*	*Rib-side distention*	*Bulimia*	Lumbago
*Bloody stool*	*Yellow fur*	Dumb	Chest, epigastric fullness, and distress	*No hard stool*

Italics represent the values correctly predicted by the model.

**Table 5:** Topics learned by LinkLDA with *K*=40.

LinkLDA				
Two deficiency syndrome of liver and kidney	Syndrome of dampness-heat blocking collaterals	Syndrome of dampness-heat diffusing downward	Syndrome of yang deficiency of spleen and kidney	Syndrome of yin deficiency and dampness-heat
Less urine volume	Depression	Thin fur	Sallow complexion	*Bulgy tongue*
Hand edema	*Weak knee*	Soreness of waist	Soreness of waist	*Thirst without desire to drink*
*No hard stool*	*Dizziness*	Hard stool	Loose stool	Irritability
*Leg swelling*	*No hard stool*	*Rib-side distention*	*Lassitude*	*Bitter taste*
Loose stool after bowel hard	Dark red tongue	*Bodily pain*	*Bulimia*	*Leg numb*
*Bloody stool*	Normal sleep	*Dark red tongue*	Lip color: purple	Brown macules on the skin
*Dark red tongue*	*Heartburn*	*Borborygmus*	*Dark red tongue*	*Yellow fur*
Chest, epigastric fullness, and distress	*Weak*	*Dumb*	*Normal urination*	*Skelalgia*
*Profuse spittle*	Palpitation	*Bowel 1 per day*	No abdominal distention	Stringy pulse
Loose stool	*Bowel 1 per day*	*Teeth-marked tongue*	*Vexation*	*No hard stool*

Italics represent the values correctly predicted by the model.

**Table 6:** Topics learned by block-LDA with *K*=40.

Block-LDA				
Two deficiency syndrome of liver and kidney	Syndrome of dampness-heat blocking collaterals	Syndrome of dampness-heat diffusing downward	Syndrome of yang deficiency of spleen and kidney	Syndrome of yin deficiency and dampness-heat
Soreness of waist	*Hard stool*	*Red tongue*	Soreness of waist	*Thin fur*
*Dark red tongue*	Dark red tongue	Rapid pulse	*Numbness of hand*	Dark red tongue
Weak	*Thin fur*	Bowel 3 per day	*Inability to walk*	*Skelalgia*
Slippery pulse	Soreness of waist	*Nausea*	*Hematuria*	*Uneven pulse*
*Skelalgia*	Yellow Fur	Normal urination	Pale complexion	Stool forming
Bowel 1 per day	No abdominal distention	No abdominal distention	*Lassitude*	Lumbago
No hard stool	*Bowel 1 per day*	Hard stool	Bowel 1 per day	Normal urination
Lip color: purple	Spiritlessness	*Dark red tongue*	Loose stool	No abdominal distention
Normal sleep	Normal diet	*Yellow fur*	Emaciation	*No hard stool*
*Yellow fur*	Normal urination	Weak	No abdominal distention	*Yellow fur*

Italics represent the values correctly predicted by the model.

**Table 7:** Topics learned by SSTM with *K*=40.

SSTM				
Two deficiency syndrome of liver and kidney	Syndrome of dampness-heat blocking collaterals	Syndrome of dampness-heat diffusing downward	Syndrome of yang deficiency of spleen and kidney	Syndrome of yin deficiency and dampness-heat
Inhibited defecation	*Knee pain*	Dumb	*Fissured tongue*	Thirst without desire to drink
Hand edema	Depression	*Dark red tongue*	Soreness of waist	Brown macules on the skin
Bulgy tongue	*Chest, epigastric fullness, and distress*	Soreness of waist	Loose stool	*Epistaxis*
Difficulty in micturition	Dark red tongue	Emaciation	No abdominal distention	Stringy pulse
*Stomachache*	Spontaneous perspiration	*Borborygmus*	*Dizziness*	Dark red tongue
*Profuse spittle*	Aversion to cold	Bloody stool	*Dark red tongue*	*Hematochezia*
Aversion to cold	*Arthralgia*	*Nausea*	*Lassitude*	*Hematuria*
*Palpitation*	Palpitation	Greenish complexion	Sallow complexion	Dumb
Chest tightness	Indigestion	*Lochiostasis*	Lip color: purple	Normal sleep
No abdominal distention	*Hand edema*	Diuresis	Turbid urine	Bowel 1 per day

**Table 8:** Topics learned by SDTM with *K*=40.

SDTM				
Two deficiency syndrome of liver and kidney	Syndrome of dampness-heat blocking collaterals	Syndrome of dampness-heat diffusing downward	Syndrome of yang deficiency of spleen and kidney	Syndrome of yin deficiency and dampness-heat
Inhibited defecation	Lumbar flaccidity	Soreness of waist	Rapid pulse	Blurred vision
Bulgy tongue	*Knee pain*	Thin fur	Sallow complexion	Stringy pulse
Less urine volume	*Weak knee*	Hard stool	Effulgent gallbladder fire	Dark red tongue
Hand edema	Bowel 1 per day	*Teeth-printed tongue*	Emaciation	Irritability
Loose stool after bowel hard	Desire for drinking	Weak	Soreness of waist	Dumb
*Leg swelling*	No swelling of the lower extremities	*Rib-side distention*	Loose stool	Thirst without desire to drink
Difficulty in micturition	No pedal edema	Dumb	*Lassitude*	Brown macules on the skin
Bowel 1 per day	Normal sleep	Normal urination	Chest, epigastric fullness, and distress	Normal diet
Normal sleep	Depression	Normal sleep	Lip color: purple	*Epistaxis*
Normal diet	Loose stool	Bowel 3 per day	Abnormal diet	Bowel 1 per day

Symptoms indicate that the patterns of TCM syndrome differentiation have high quality.

## Data Availability

The authors collected 1959 medical records on CKD from Beijing Dongzhimen Hospital, which include 948 (48.4%) females and 1011 (51.6%) males only to support the research work. Because these records involve the patients' privacy information, the authors have not obtained the authorization of the hospital. Therefore, the authors cannot publish them on the Internet for public sharing at present.
